# *lncRNA260* siRNA Accelerates M2 Macrophage Polarization and Alleviates Oxidative Stress via Inhibiting *IL28RA* Gene Alternative Splicing

**DOI:** 10.1155/2022/4942519

**Published:** 2022-09-23

**Authors:** Xin-Xing Yang, Yan-Yan Li, Ge Gong, Hong-Yu Geng

**Affiliations:** ^1^Department of Gerontology, First Affiliated Hospital of Nanjing Medical University, Nanjing, China; ^2^Department of Intensive Care Unit, Affiliated Hospital of Yangzhou University, Yangzhou, China; ^3^Clinical Research Center, First Affiliated Hospital of Nanjing Medical University, Nanjing, China; ^4^Department of Gerontology, General Hospital of Eastern Theater Command, Nanjing, China; ^5^Department of Intensive Care Unit, Baoding First Central Hospital, Baoding, China

## Abstract

The macrophage transformation of inflammatory M1 to anti-inflammatory M2 could be promoted by activating PI3K/AKT signaling pathway. In our previous study, it was found that downregulation of lncRNA260 could ameliorate hypoxic cardiomyocyte injury by regulating IL28RA through the activation of PI3K/AKT signaling pathways. It was suggested that lncRNA260 siRNA could promote the macrophages toward M2 polarization by regulating *IL28RA*. In this study, lncRNA260 siRNA was used to observe its effect on the polarization of murine bone marrow-derived macrophages (BMDM) and investigate its related mechanisms. lncRNA 260 specific siRNA were designed and synthesized which were transfected into murine BMDM with liposomes. The experiment was divided into three groups: Hypoxia group, Hypoxia+lncRNA 260-specific siRNA transfection group, and Normoxia group. The CD206-APC/CD11b-FITC or CD206-FITC/CD107b (Mac-3) double positive proportions were used to compare the M2 polarization proportions in the hypoxia process by using the immunofluorescence staining method. The p-AKT, Arg 1, PI3KCG, IL28RAV1, and IL28RAV2 protein expression changes were observed by using the western blot method. Compared with the Normoxia group, the M2 proportions were significantly decreased in the Hypoxia group (*P* < 0.05). Compared with the hypoxia group, the M2 proportions were significantly increased in the Hypoxia+lncRNA260 siRNA transfection group (*P* < 0.05). In the Hypoxia group, the ratios of Arg 1/*β*-Actin, p-AKT/*β*-Actin, PI3KCG/*β*-Actin, and IL28RAV1/*β*-Actin were significantly lower than those in the Normoxia group (*P* < 0.05). After transfection with lncRNA260 siRNA, the ratios of Arg1/*β*-Actin, p-AKT/*β*-Actin, PI3KCG/*β*-Actin, and IL28RAV1/*β*-Actin were significantly higher than those in the Hypoxia group (*P* < 0.05). Compared with the Normoxia group, the IL28RAV2/*β*-Actin in the Hypoxia group was significantly increased (*P* < 0.05). After transfection with lncRNA260 siRNA, the ratio of IL28RAV2/*β*-Actin was significantly decreased than that in the Hypoxia group (*P* < 0.05). lncRNA260 siRNA could promote the M2 polarization of the hypoxia macrophages by reducing the IL28RAV2 alternative splicing variant, which might be related to the activation of the JAK-STAT and PI3K/AKT signaling pathways. It will provide a new strategy for the anti-inflammation, antioxidative stress therapy, and cardiac remodeling after AMI.

## 1. Introduction

Acute myocardial infarction (AMI) is a major disease that is threatening people's health nowadays. The progress of intervention and drug therapy has also brought great improvement in the treatment of AMI. However, cardiac remodeling is a major cause of death in AMI patients. Therefore, cardiac remodeling is an urgent problem to be solved. Cardiac remodeling after myocardial infarction is a process of changes in cardiac geometry and function, and it is considered to be a common response to increased ventricular wall adaptability or reduced viable myocardium. Cardiac remodeling would lead to the impaired cardiac function and even heart failure. In the early stage of AMI, inflammation and immune response occur to limit the ischemic infarct size and maintain cardiac output. However, excessive and long-term inflammation aggravates ventricular remodeling after AMI.

During AMI, acute myocardial ischemia, hypoxia, impaired mitochondrial function, and activation of neutrophils increase oxygen free radicals. Oxidative stress activates the inflammatory gene promoter of monocytes through the nuclear factor KB pathway, and then, the related mRNA activates transcription to produce inflammatory factors. In turn, inflammatory factors generate reactive oxygen species through the oxidation of NADPH oxidase complexes on the white cell membrane to amplify the reaction of oxidative stress and further stimulate the activation of inflammatory cells. Therefore, oxidative stress and inflammatory reaction form a vicious spiral [1, 2]. The process of AMI is the oxidative stress process in which prooxidation dominates, and it interacts with and influences the inflammatory response. Thus, it further strengthens the chain reaction between oxidation and inflammation. These phenomena jointly lead to the occurrence and progression of AMI. Therefore, alleviating inflammatory response after AMI could reduce oxidative stress and promote myocardial repair after infarction [3].

Macrophage is an important component of inflammation and plays an important role in later heart remodeling. M1 and M2 macrophages play different roles in the inflammatory stage and myocardial remodeling after infarction. The early stage of inflammation is dominated by M1 type, which secretes proinflammatory cytokines and promotes the development of inflammation. M2 type is dominant in the late stage of inflammation, and it promotes inflammation subsidence, proliferation of fibroblasts, and formation of new vessels. According to the previous studies, the expression of monocyte chemotaxis protein-1 was gradually upregulated within 3 days after AMI in mice, and it reached its peak on the third day. After AMI, the secretion of inflammatory factors and cytokines gradually increased, which attracted a large number of macrophages. The recruited M1 macrophages and other inflammatory cells secreted a large number of cytokines and chemokines, which recruited more inflammatory cells. The M1 macrophages decreased after AMI three days, and the M2 macrophages increased and participated in cardiac remodeling by secreting anti-inflammatory cytokines; these phenomena promoted the formation and proliferation of myofibroblasts and new vessels [4]. The imbalance of M1 and M2 macrophages during inflammation will lead to poor ventricular remodeling. Therefore, the therapy targeting M1/M2 macrophage transformation can inhibit early inflammation and promote late cardiac repair. This way effectively blocks cardiac remodeling after AMI.

Interleukin-28 receptor *α* (IL28RA) and IL10RB constitute the receptors of type III interferon (IFN-*λ*s). Type III interferon is a new type of interferon, which belongs to the IL10 family of class II cytokines. IL28RA is widely present in various tissues of the human body, and it is highly expressed in organ tissues such as the heart, bone marrow, pancreas, thyroid, skeletal muscle, prostate, and testis [5]. Studies have shown that IFN-*λ*s can activate JAK-STAT and PI3K/AKT signaling pathways to play antiviral, antitumor proliferation roles and regulate inflammatory responses [6–11]. IL28RA has two alternative splicing (AS) variants in macrophages, namely, IL28RAV1 and IL28RAV2; the two variants can bind to type III interferon, but IL28RAV2 loses the signal transduction function and can inhibit the activity of IFN-*λ*s; thus, they have opposite functions [11, 12]. The M2-type polarization of macrophages is related to the activation of JAK-STAT and PI3K/AKT signaling pathways, which promote the transformation of macrophages from the inflammatory M1-type to the anti-inflammatory M2-type [12–14]. Different IL28RA AS variants promote different phenotypic transformation of macrophages. IL28RAVl promotes M2-type polarization of macrophages, while IL28RAV2 inhibits this function.

Our previous studies have shown that downregulation of lncRNA260 regulates IL28RA and activates the JAK-STAT and PI3K/AKT signaling pathways, and this phenomenon improves the injury of hypoxic cardiomyocytes in rats [15]. This effect is thought to be related to the reduction in IL28RAV2. Therefore, we speculate that lncRNA260-specific siRNA could reduce the expression of *IL28RAV2* gene, activate JAK-STAT and PI3K/AKT signaling pathways, promote the polarization of macrophages to M2-type, inhibit inflammatory response, and thus achieve certain biological effects.

This study was performed to verify the abovementioned hypothesis. Here, lncRNA260-specific siRNA was designed and transfected into murine bone marrow-derived macrophages (BMDM) with liposome transfection method for hypoxia intervention to explore the effect and related mechanism of macrophage polarization in hypoxia model.

## 2. Materials and Methods

### 2.1. Materials

The following were used in the study: collagenase and Dulbecco Modified Eagle medium (DMEM) cell culture medium (Gibco, USA), Lipofectamine™ 2000 (Invitrogen, USA), IL28RA rabbit antibody (Sigma, USA), FITC rat anti-mouse CD206 (MMR) antibody (Biolegend, USA), APC rat anti-mouse CD206 (MMR) antibody (Biolegend, USA), FITC rat anti-mouse CD11b antibody (Biolegend, USA), rat anti-mouse CD107b (Mac-3) antibody (Biolegend, USA), *β*-Actin rabbit antibody (Cell Signaling, USA), phospho-AKT (pAKT) (Ser 473) rabbit antibody (Cell Signaling, USA), Arginase 1 (Arg 1) goat antibody (Santa Cruz, USA), PI3KCG mouse antibody (Santa Cruz, USA), Donkey F (ab)2 Anti-Rat IgG H&L(Alexa Fluor® 568) preadsorbed (Abcam, UK), peroxidase-conjugated AffiniPure rabbit anti-goat IgG(H+L) (Jackson, USA), goat anti-rabbit IgG-HRP (Absin Bioscience Inc., China), and peroxidase-conjugated AffiniPure goat anti-mouse IgG(H+L) (ZSGB-BIO, China).

The healthy C57BL/6 mice (6-8 weeks old, 16-20 g weight) were from the Jiangsu Province Animal Center. The lncRNA260-specific siRNA was synthesized by Shanghai Gene Pharma Co., Ltd. The nucleotide sequence is listed in Table 1.

### 2.2. Methods

#### 2.2.1. Mononuclear Macrophages from Murine Bone Marrow Isolation and Culture [16]

The current research was approved by the Ethics Committee of the First Affiliated Hospital of Nanjing Medical University (No. 2021-SRFA-007). C57BL/6 mice were sacrificed by using CO_2_ inhalation in a rodent euthanasia device. Their hind limbs were cut off and placed in petri dishes containing sterile PBS and moved to a super-clean platform. The hind limbs were rinsed with PBS twice, and the muscles of the hind limbs were removed successively. The hind limbs were rinsed with PBS again 1-2 times and then placed in a small amount of PBS. The ends of the thigh and tibia were cut open at the joint, and PBS was absorbed with a 1 mL syringe to rinse the bone marrow cavity until it turned white. Bone marrow rinses were collected and filtered through a 200-mesh filter. The bone marrow cells were centrifuged at room temperature at 300 g for 5 min, and the supernatant was discarded.

After cell counting, an appropriate amount of DMEM was added and the final concentration of cell suspension was adjusted to 1 × 10^6^ cells/mL. The cells were inoculated in 24-well plates, 6-well plates, and 3.5 cm petri dishes. On the third day, the experiment was randomly divided into groups. The experiment was divided into three groups: Hypoxia+lncRNA260 siRNA transfection group, Hypoxia group, and normal control group (Normoxia group).

#### 2.2.2. Transfection of Murine BMDM with lncRNA260 siRNA

After culturing murine BMDM for 3 days, penicillin/streptomycin was removed from the DMEM culture medium and lncRNA260 siRNA were transfected into the cells at the 100 nmol/L concentration by Lipofectamine transfection method. In each group, triplicate parallel wells were set up. After the Lipofectamine 2000 was dissolved in DMEM medium and mixed with lncRNA260 siRNA, the Lipofectamine-lncRNA260 siRNA mixture was added into the mononuclear macrophages culture wells, respectively, and gently blended. After transfection for 4 hours at 37°C in the incubator, the Lipofectamine 2000 was removed. The culture medium was then changed with new complete DMEM medium containing penicillin/streptomycin.

#### 2.2.3. Establishing the Murine BMDM Hypoxia Model

72 hours after BMDM transfection, all groups except controls were treated with hypoxia for 24 hours by using Anaerobic bag (Becton Dickinsonand Inc., USA) (95% N_2_ and 5% CO_2_) to simulate the Hypoxia process.

#### 2.2.4. Measuring CD107b(Mac-3), CD11b, and CD206 proteins Expression in Cultured Murine BMDM by Immunofluorescence Staining

After the hypoxia process, the 24-well cell plate was removed from the hypoxia bag and rinsed with PBS 2-3 times. 4% paraformaldehyde (PFA) was added to each well and fixed at room temperature (RT) for 15 min and rinsed with PBS 3 times. 0.2%triton was added to each well, and the triton was permeated at RT for 5 min. After Triton was discarded and the wells were rinsed with PBS for 3 times, 3% normal lamb serum (3% in PBS) was added. After the cells were blocked at RT for 1 h, the serum was discarded. The antibodies CD11b-FITC, Mac-3 and CD206-APC, and CD206-FITC were diluted with 3% lamb serum at a ratio of 1 : 100. The cells were double stained with the CD11b-FITC, CD206-APC, Mac-3, and CD206-FITC antibodies, respectively. 3% lamb serum containing antibodies were added into each well and incubated overnight at 4°C dark for more than 18 h. Then, the wells were rinsed with PBS for 3 times. Alexa Fluor® 568-conjugated donkey anti-rat IgG (H+L) antibody was diluted with 3% lamb serum at the ratio of 1 : 500. The diluted fluorescent secondary antibody was added to each well and incubated for 1 h at RT, away from light. Then, the wells were rinsed with PBS for 4 times. The 4′,6-diamidino-2-phenylindole (DAPI) dyeing solution was added to each well. The anti-fade fluorescence mounting medium was dropped on the slide. Then, the slide was removed from the wells and covered back on the glass slide. The macrophage glass slides were observed under the fluorescent microscope (Olympus, Japan) and photographed.

#### 2.2.5. Measuring proteins Expression of Cultured Murine BMDM by Western Blot

The phenylmethylsulfonyl fluoride (PMSF) : RIPA lysis buffer was prepared in a ratio of 1 : 100 for full protein extraction lysis buffer. The total protein was extracted from cultured murine BMDM by using this RIPA lysis buffer. The total protein was quantified by using Bicinchoninic acid method. The total protein was separated through 10% SDS-PAGE electrophoresis. Then, they were transferred to polyvinylidene fluoride (PVDF) membrane. The transferred PVDF membrane was blocked overnight at 4°C by using the 5% skim milk. The 1 : 1000 diluted primary antibodies (goat anti-mouse Arg 1 antibody, rabbit anti-mouse IL28RA antibody, rabbit anti-mouse *β*-Actin antibody, rabbit anti-mouse pAKT antibody, and mouse anti-mouse PI3KCG antibody) were incubated with the proteins on the shaker at 4°C overnight. The horseradish peroxidase-labeled secondary antibodies (rabbit anti-goat IgG antibody, goat anti-rabbit IgG antibody, and goat anti-mouse IgG antibody) were diluted at a ratio of 1 : 5000 and incubated with the proteins on the shaker for 2 hours at 4°C. The Thermo Scientific pierce Super Signal West Femto Chemiluminescent Substrate was used to develop the antibodies incubated PVDF membrane for 1 min. After the PVDF membrane was washed in the double-distilled water, it was exposed and photographed with the Gel Imaging System. The optical density of the proteins was calculated and compared.

### 2.3. Statistical Analysis

SPSS23.0 statistical software was used for statistical analysis. The Kolmogorov-Smirnov test was used to examine whether the measurement data conform to the normal distribution or not. If the measurement data conform to the normal distribution, they were expressed as the mean ± standard deviation. A *t*-test was used for the comparison of measurement data between the two groups. Otherwise, a rank sum test would be used. One-way ANOVA was used for the comparison between multiple groups. *P* < 0.05 indicated that the difference was statistically significant.

## 3. Results

### 3.1. The M2 Murine BMDM Proportion Changes during the Hypoxia Process by Immunofluorescence Method

#### 3.1.1. Culture of BMDM from Adult C57BL/6 Mice

The nonadherent cells of murine BMDM just extracted were found to be round under the microscope. After 48 hours of culture, the adherent cells were observed to be round or irregular under the microscope, with pseudofoot protrusion, and the cell size was basically uniform (Figures 1(a) and 1(b)).

#### 3.1.2. The CD11b and CD206 proteins Localization and Relative Levels by Immunostaining in the Murine BMDM Hypoxia Process

CD107b (Mac-3) and CD11b are mainly expressed in all macrophage populations, and CD206 is a specific surface marker of M2-type macrophages. DAPI staining is the nucleus. Compared with the normal group (0.45 ± 0.04), the double positive proportion of CD206/CD11b was decreased in the hypoxia group (0.26 ± 0.01) (*P* < 0.05). Compared with the hypoxia group, the CD206/CD11b double positive double positive proportion (0.80 ± 0.04) was significantly increased in the Hypoxia+lncRNA260 siRNA transfection group (*P* < 0.05) (Figures 2(a) and 2(b)).

#### 3.1.3. The Mac-3 and CD206 proteins Localization and Relative Levels by Immunostaining in the Murine BMDM Hypoxia Process

Compared with the normal group (0.48 ± 0.04), the double positive proportion of CD206/Mac-3 was decreased in the hypoxia group (0.28 ± 0.01) (*P* < 0.05). Compared with the hypoxia group, the CD206/CD11b double positive proportion (0.81 ± 0.04) was significantly increased in the Hypoxia+lncRNA260 siRNA transfection group (*P* < 0.05) (Figures 3(a) and 3(b)).

### 3.2. The Expression Changes of Arg 1, p-AKT, and PI3KCG Proteins in the Murine BMDM Hypoxia Process Detected by Western Blot

After transfection of lncRNA260 siRNA into murine BMDM for 72 h and 24 h hypoxia intervention, the expression of Arg 1, p-AKT, and PI3KCG proteins was detected by Western blot, and the expression changes of Arg 1, p-AKT, and PI3KCG proteins were compared. All of them were statistically analyzed by the grayscale ratio with internal reference *β*-Actin (Figure 4(a)).

Arg 1 protein is one of the characteristic proteins of M2 macrophages. In the Hypoxia group, the ratios of Arg 1/*β*-Actin, Arg 1/*β*-Actin, PI3KCG/*β*-Actin were 0.81 ± 0.05, 0.67 ± 0.01, and 0.62 ± 0.01, respectively, which were significantly lower than those in the Normoxia group (1.00 ± 0.01) (*P* < 0.05). After transfection with lncRNA260 siRNA, the ratios of Arg1/*β*-Actin, p-AKT/*β*-Actin, and PI3KCG/*β*-Actin were increased to 1.65 ± 0.03, 2.30 ± 0.03, and 1.03 ± 0.02 which were significantly higher than those in the Hypoxia group (*P* < 0.05) (Figure 4(b)).

### 3.3. The Expression Changes of IL28RAV1 and IL28RAV2 Proteins in the Murine BMDM Hypoxia Process Detected by Western Blot

The protein gray levels of IL28RAV1/*β*-Actin and IL28RAV2/*β*-Actin were both based on the Normoxia group. Compared with the Normoxia group, the ratio of IL28RAV1/*β*-Actin in the Hypoxia group was significantly decreased (1.00 ± 0.01 vs. 0.59 ± 0.01, *P* < 0.05). After transfection with lncRNA260 siRNA, the ratio of IL28RAV1/*β*-Actin was significantly higher than that in the Hypoxia group (0.90 ± 0.02 vs. 0.59 ± 0.01, *P* < 0.05). Compared with the Normoxia group, the IL28RAV2/*β*-Actin in the Hypoxia group was significantly increased (1.00 ± 0.01 vs. 1.31 ± 0.03, *P* < 0.05). After transfection with lncRNA260 siRNA, the ratio of IL28RAV2/*β*-Actin was significantly decreased than that in the Hypoxia group (0.82 ± 0.02 vs. 1.31 ± 0.03, *P* < 0.05) (Figures 5(a) and 5(b)).

## 4. Discussion

In this study, the M2 murine BMDM proportion was significantly decreased in the hypoxia process (*P* < 0.05). After transfection with lncRNA260 siRNA, the proportion of M2 murine BMDM was significantly increased (*P* < 0.05). Meanwhile, the proteins expression of the Arg 1, p-AKT, PI3KCG, and IL28RAV1 changed in the same way as the proportion of M2 murine BMDM. Conversely, the IL28RAV2 protein expression presented the changes in the opposite direction in the murine BMDM hypoxia process. Notably, lncRNA260 siRNA could promote the M2 polarization of the hypoxia murine BMDM by reducing the IL28RAV2 AS variant. This performance might be related to the activation of the JAK-STAT and PI3K/AKT signaling pathways.

CD206 is considered to be one of the markers of M2 macrophages. The factors inducing CD206 expression include the following: IL-4, IL-13, M-CSF, IL-10, IL-6, and glucocorticoids. However, TNF-alpha, TGF-beta, IFN-gamma, and LPS have been reported to downregulate CD206 expression. Hence, CD206 high expression is a characteristic marker of M2 macrophages. Considering only a small fraction of CD206 is present at the cell surface, intracellular staining was performed in the current research. Since all of the macrophages could express CD11b and Mac-3, the combination of CD206/CD11b or CD206/Mac-3 antibodies was respectively used to detect these proteins and the double positive expression represented these cells were M2 macrophages.

The degree of inflammation after AMI is positively correlated with the size of myocardial infarction, but the research on blocking inflammation has not obtained ideal results [17–24]. Moderate suppression of inflammatory storm after AMI could reduce myocardial injury and improve prognosis. Meanwhile, blocking the inflammatory process was not conducive to myocardial repair, and it increased the risk of pathological cardiac remodeling and cardiac rupture. The latest evidence for anti-inflammatory therapy after AMI is available. After PCI treatment of AMI, anti-inflammatory treatment with colchicine could reduce infarct size and improve prognosis [25]. Intravenous application of metoprolol after AMI could reduce the inflammatory response and limit the infarct size by reducing neutrophil tissue infiltration and its interaction with platelets in myocardial infarction area [26].

Peripheral blood mononuclear macrophages are recruited into damaged myocardium after AMI. This process is critical for cardiac repair because they could adopt proinflammatory or repair phenotypes to regulate inflammatory or repair responses, respectively [27, 28]. M1 type macrophage was dominant first and then reached the peak on 3–4 days after AMI. This phenomenon mainly produced inflammatory cytokines (e.g., TNF-*α*, IL-1*β*, and IL-6) and chemokines (e.g., CCR2, CXCL1, and IL-8), which aggravated the degree of inflammation and oxidative stress. Then, after entering the fiber proliferation stage, Arg 1, IL-10, VEGF, and TGF-*β*1 were mainly produced, and necrotic cells were cleared through cell burial [29, 30]. Furthermore, inflammation was inhibited, neovascularization was promoted, and damaged tissue repair was promoted. The peak value was reached on 6-7 days after AMI. Finally, cardiac remodeling, or scar formation, occurred, and the necrotic areas of the myocardium were replaced by fibrous scar tissue formed by cross-linked fibers. The early stage of inflammatory response after AMI is a critical time for cardiac remodeling. Thus, finding genes or drugs that can promote the macrophage phenotype from proinflammatory M1 to anti-inflammatory M2 is important. The transformation from inflammatory M1 type macrophages to anti-inflammatory M2 type could be accelerated by activating PI3K/AKT signaling pathway [13, 14]. In our previous study, we found that downregulation of lncRNA260 could ameliorate hypoxic cardiomyocytes injury by regulating IL28RA through the activation of PI3K/AKT signaling pathways. lncRNA260 siRNA could also promote the macrophages toward M2 polarization by regulating IL28RA.

Studies have shown that IL28RA has various alternative spliceosomes with different functions [12]. IL28RAV1 is a normal functioning CRF2-12. IL28RAV2 lacks 29 amino acids in the intracellular region and can bind to type III interferon, but it loses the signal transduction function. IL28RAV2 can inhibit the activity of IFN-*λ*1, and it is a negative regulator of type III interferon, which plays an anti cell proliferation and promotes inflammatory response. In the current study, murine BMDM also expressed two AS variants, namely, 59KD and 55KD. After 24 h hypoxic exposure, the full length of 59KD IL28RAV1 was significantly reduced, and the expression of 55KD IL28RAV2 was significantly increased. This finding is speculated to be related to IL28RA mRNA AS caused by hypoxia, which inhibits JAK-STAT and PI3K/AKT signaling pathways, promotes polarization of macrophages to M1, enhances inflammatory response and oxidative stress, significantly increases apoptosis and necrosis of myocardial cells, and increases the risk of myocardial fibrosis and heart rupture. After lncRNA260 siRNA intervention, the IL28RAV2 AS was significantly reduced and IL28RAV1 was significantly increased compared with that of the hypoxia group. These phenomena promoted the activation of JAK-STAT and PI3K/AKT signaling pathways, caused the M2 polarization of macrophages, and reduced the inflammatory response. IL10RB is a common receptor ligand of IL28RA and IL10RA. During AMI, the expression of IL28RAV2 is upregulated in macrophages, which results in a competitive increase in the heterodimer formed by IL10RB and IL28RAV2. Meanwhile, the binding of IL10RA receptor is reduced. When hypoxia occurs, the expression of IL10RA is downregulated due to the inhibition of type III interferon signaling pathway. This phenomenon further reduces the activation of IL10/STAT3/IL4RA/STAT6, decreases M2 macrophages, further reduces the secretion of IL10, and aggravates inflammation.

catRAPID omics is a server for large-scale calculations of protein-RNA interactions [31].

The catRAPID omics predicted that lncRNA260 could competitively bind to the SF3B2 and SF3B3 splicing complex with IL28RA. The ESE finder predicts that lncRNA260 also has the exon splicing enhancer (ESE) sequence of the SRSF protein recognition site of the splicing enhancer, which competitively binds to the SRSF protein with IL28RA (http://krainer01.cshl.edu/cgi-bin/tools/ESE3/esefinder.cgi?process=home) [32, 33]. Thus, it affected the recognition and splicing of the 7^th^ exon of IL28RA mRNA by the splicing body, resulting in partial loss of the 7^th^ exon, and increased the IL28RAV2 AS variant.

In contrast to IL28RAV1, this IL28RAV2 variant blocked JAK-STAT and PI3K/AKT signaling pathways, resulting in decreased M2-type polarization of macrophages and enhanced inflammatory response, leading to myocardial cell damage and ventricular remodeling during AMI.

## 5. Conclusion

In a word, lncRNA260 siRNA could promote M2 macrophage polarization and alleviate oxidative stress by inhibiting IL28RAV2 AS in the murine BMDM hypoxia process. Considering the current study is an in vitro experiment, this conclusion will be further confirmed in the animal experiments. This study will lay a foundation for future in vivo research. A preprint has previously been published [34].

## Figures and Tables

**Figure 1:** The morphological characteristics of murine BMDM. Under the microscope, the murine BMDM were round or irregular, with pseudofoot protrusion, and the cell size was basically uniform. (a) The normal cell shape under 100x magnification. (b) The normal cell shape under 200x magnification.

**Figure 2:** The CD11b and CD206 proteins localization and relative levels by an immunostaining method in the murine BMDM hypoxia process. (a) The M2 macrophage changes during the hypoxia process by an immunofluorescence method. In the CD11b-FITC and CD206-APC double staining group, green was positive CD11b-FITC, red was positive CD206-APC, and blue was DAPI staining. The scale in each picture means 100 *μ*m. (b) The M2 macrophage proportion changes during the hypoxia process. ^∗^*P* < 0.05, compared with the Hypoxia group; ^△^*P* < 0.05, compared with the normal control group.

**Figure 3:** The Mac-3 and CD206 proteins localization and relative levels by immunostaining in the murine BMDM hypoxia process. (a) The M2 macrophage changes during the hypoxia process by an immunofluorescence method. In Mac-3 and CD206-FITC double staining group, green was positive CD206-FITC, red was positive Mac-3, and blue was DAPI staining. The scale in each picture means 100 *μ*m. (b) The M2 macrophage proportion changes during the hypoxia process. ^∗^*P* < 0.05, compared with the Hypoxia group; ^△^*P* < 0.05, compared with the normal control group.

**Figure 4:** The expression changes of Arg 1, p-AKT, and PI3KCG proteins detected by Western blot in the murine BMDM hypoxia process. (a) The western blot developing figure for the Arg 1, p-AKT, and PI3KCG proteins in the murine BMDM hypoxia process. (b) The ratio changes of Arg 1/*β*-Actin, p-AKT/*β*-Actin, and PI3KCG/*β*-Actin were detected by Western blot in the murine BMDM hypoxia process. ^∗^*P* < 0.05, compared with the Hypoxia group; ^△^*P* < 0.05, compared with the normal control group.

**Figure 5:** The expression changes of IL28RAV1 and IL28RAV2 proteins detected by Western blot in the murine BMDM hypoxia process. (a) The Western blot developing figure for the IL28RAV1 and IL28RAV2 proteins in the murine BMDM hypoxia process.  Figure 5(b). The ratio changes of IL28RAV1/*β*-Actin and IL28RAV2/*β*-Actin were detected by Western blot in the murine BMDM hypoxia process. ^∗^*P* < 0.05, compared with the Hypoxia group; ^△^*P* < 0.05, compared with the normal control group.

**Table 1:** The nucleotide sequence of lncRNA260-specific siRNA.

siRNA	Nucleotide sequence
Sense chain	5′-CCCAGUGAAGGAGACGAAATT-3′
Antisense chain	5′-UUUCGUCUCCUUCACUGGGTT-3′

## Data Availability

All data generated or analyzed during this study are included in this article. Further enquiries can be directed to the corresponding author.
